# Serum levels of preS antigen (HBpreSAg) in chronic hepatitis B virus infected patients

**DOI:** 10.1186/1743-422X-4-93

**Published:** 2007-09-24

**Authors:** Min Lian, Xu Zhou, Lai Wei, Shihong Qiu, Tong Zhou, Lanfen Li, Xiaocheng Gu, Ming Luo, Xiaofeng Zheng

**Affiliations:** 1 National Laboratory of Protein Engineering and Plant Genetic Engineering, Peking University, Beijing, 100871, China; 2 Department of Biochemistry and Molecular Biology, College of Life Sciences, Peking University, Beijing, 100871, China; 3 Department of Microbiology, University of Alabama at Birmingham, Birmingham, Alabama, 35294, USA; 4 Department of Medicine, University of Alabama at Birmingham, Birmingham, Alabama, 35294, USA; 5 Peking University People's Hospital, Beijing, 100014, China

## Abstract

**Background:**

Hepatitis B virus (HBV) infection is a serious health problem worldwide. Treatment recommendation and response are mainly indicated by viral load, e antigen (HBeAg) seroconversion, and ALT levels. The S antigen (HBsAg) seroconversion is much less frequent. Since HBeAg can be negative in the presence of high viral replication, preS antigen (HBpreSAg) might be a useful indicator in management of chronic HBV infection.

**Results:**

A new assay of double antibody sandwich ELISA was established to detect preS antigens. Sera of 104 HBeAg-negative and 50 HBeAg-positive chronic hepatitis B patients have been studied and 23 HBeAg-positive patients were enrolled in a treatment follow-up study. 70% of the HBeAg-positive patients and 47% of the HBeAg-negative patients showed HBpreSAg positive. Particularly, in the HBeAg-negative patients, 30 out of 47 HBpreSAg positive patients showed no evidence of viral replication based on HBV DNA copies. A comparison with HBV DNA copies demonstrated that the overall accuracy of the HBpreSAg test could reach 72% for active HBV replication. HBpreSAg changes were well correlated with changes of HBsAg, HBV DNA and ALT levels during the course of IFN-α treatment and follow-up. HBeAg positive patients responded well to treatment when reduction of HBpreSAg levels was more pronounced.

**Conclusion:**

Our results suggested that HBpreSAg could be detected effectively, and well correlated with HBsAg and HBV DNA copies. The reduction of HBpreSAg levels in conjunction with the HBV DNA copies appears to be an improved predictor of treatment outcome.

## Background

Hepatitis B virus (HBV) disease continues to be an important health problem worldwide. Estimated 360 million people are chronically infected by HBV and new chronic cases continue to accumulate [1]. Long-term treatment with interferon and/or nucleoside analog drugs will be required for these patients [2-4]. It is therefore valuable to have clinical indicators that support the optimal treatment of HBV infection. In addition, drug resistant mutants and genotypic variants should also be monitored.

Chronic HBV patients are classified in three states: inactive HBsAg carrier-state, HBeAg-positive, and HBeAg-negative chronic hepatitis B. The inactive HBsAg carrier-state is characterized by the presence of HBsAg and anti-HBe, normal aminotransferase (ALT) level and low or undetectable level of HBV DNA in serum, indicating that HBV replication may be suppressed in the carriers. In the other two states, HBV DNA can be detected at a much higher level in HBeAg-positive chronic hepatitis B patients than that in HBeAg-negative chronic hepatitis B patients. Therefore, treatment is usually recommended for the HBeAg-positive chronic HBV patients and the endpoint is measured typically by loss of HBeAg and low levels of HBV DNA (<10^5 ^copies/ml) in serum[5]. In addition, ALT level is also referenced in recommendation for antiviral therapy[6]. However, the number of HBeAg-negative, anti-HBe positive, and high DNA copies (>10^4^-10^5 ^copies/ml) hepatitis B is increasing, especially in Asia and Southern Europe[7], and many cases of these patients relapsed and caused liver cirrhosis and hepatocellular carcinoma. Treatment regiments for these cases need to be altered based on more appropriate predictors. Demonstration of clinical efficacy for HBeAg-negative cases with new drugs also requires alternative markers, not only to indicate virus replication but also to predict anti-virus response besides HBV DNA.

There are three surface structural proteins in HBV: Large (L), middle (M), and small (S) proteins. All three proteins contain the surface antigen (S) (226 amino acids), while an N-terminal extension of S by 55 amino acids (designated as preS2) results in the M protein (281 amino acids). The L protein has an additional preS1 domain that contains 119 (genotypes A and C) or 108 (genotype D) N-terminal amino acid residues compared to the M protein. Full length preS is composed of preS1 and preS2 (174 amino acids for genotypes A and C, or 163 for genotype D). Though HBsAg has been widely used as clinical markers, HBV surface antigen preS and its antibodies are not commonly employed. However, preS is primarily present in the DNA-containing full HBV particle as well as empty filaments [8] and it has been shown to be associated with virus attachment to the host cell receptor and membrane fusion during entry[9]. Neutralizing epitopes have been mapped in preS[10]. This special antigen also contributes to clinical application. PreS1 and preS2 peptides have been included in new formation of HBV vaccines to supplement the widely used S-based vaccines [11-13]. In some reports, preS1 or preS2 was included as serological markers in prognosis [14-18]. Nonetheless, using antibodies against full length preS containing both preS1 and preS2 to detect the serum HBpreSAg has not been reported so far. Since the functional 3D structure formed by the full length preS is the structural basis for displaying epitopes that are present on the active Dane viral particles, assays using antibodies derived from a well folded preS can result in a more accurate detection of preS antigens in serum, which is a prerequisite for improving the assay accuracy and exploitation of the potential significance of HBpreSAg as a serological indicator for HBV infection. Therefore, this study is carried out to develop a novel assay for HBpreSAg and evaluate the potential significance of serum HBpreSAg levels in management of HBV infection.

## Results

### A double antibody sandwich ELISA for measuring serum HBpreSAg

The purified polyclonal anti-preS was examined by western blot. The result showed that the polyclonal anti-preS can specifically identify the recombinant preS from *E. coli *(data not shown).

Since the amount of spheres viral particles containing HBsAg is much more than that of infectious Dane particles (infectious particles containing L-M-S antigens and viral DNA) containing full length preS antigen[19], the content of HBpreSAg in serum is more difficult to be detected effectively than HBsAg. Meanwhile, abundance of HBsAg could produce interference with assay of HBpreSAg. The following experiments were carried out to circumvent HBsAg bias.

First, a serial dilution of known amounts of recombinant S proteins was used to plot a standard curve. The amount of HBsAg present in serum was determined according to the amount of recombinant S protein. The result shown in Fig. 1B indicated that the recombinant S peptide (white square) and HBsAg (black square) in patient serum exhibited the same pattern by standardized anti-HBs antibody, which also suggested that the recombinant S protein indeed folded in the proper way compared to native HBsAg. Second, known amount of recombinant S protein was applied in anti-preS coated plates instead of serum HBsAg to examine the bias on the measurement of HBpreSAg (Fig. 1B). HBsAg has an extremely low binding affinity to the polyclonal anti-preS antibody (white circle). Serum samples exhibited a sharp increase of HBpreSAg binding to polyclonal anti-preS (black circle) before HBsAg could bring any interference based on the absorbance measurements using recombinant S protein. Thus when it is below 20 μg/ml, HBsAg would not interfere with the detection of HBpreSAg in the system analyzed. Polyclonal anti-preS can specifically capture HBpreSAg and the level of serum HBpreSAg can be examined quantitatively by this assay.

**Figure 1:** (A) A SDS-PAGE showing the purified recombinant preS. (B) Binding of HBsAg to anti-HBs and to polyclonal anti-preS. An ELISA Kit for HBsAg detection was used to detect HBsAg in the serum sample of an HBeAg positive patient (black square). Recombinant S protein (white square) was used as control. Binding of HBsAg to polyclonal anti-preS (white circle) was detected by adding recombinant S protein to a 96-well microplate which was coated with the polyclonal anti-preS antibody, using the same HRP-anti-HBs in the HBsAg kit. The binding to polyclonal anti-preS by antigens in an HBeAg positive patient serum sample is shown as (black circle). The X axis is plotted in logarithm. The absorbance at 450 nm has been subtracted by the background.

### Enhanced sensitivity in detecting preS than preS1

Full lengthpreS, other than preS fragments such as preS1, can form a well folded, functional three dimensional structure, which is the basis for displaying epitopes in native preS and a potential for detecting active Dane viral particles. Therefore, antibodies prepared against full length preS should detect well folded full length preS with greater sensitivity than fragments of preS. In order to verify this notion, both recombinant preS1 and full length preS were detected and compared. 0.1 ng of preS could be easily detected, while the same amount of preS1 presented a negative reading. The detection limit of preS1 by this ELISA is 10 ng (Fig. 2). This result indicated that full length preS can be detected much more effectively, which could be interpreted that full length preS Ag could present epitopes that were more readily recognized.

**Figure 2:** Comparison of the binding ability of preS and preS1 to anti-preS by ELISA test. Different amounts of recombinant preS1 (white square) and preS (black square) proteins (0, 0.1 ng, 1.0 ng, 10 ng and 100 ng) were added to the polyclonal anti-preS coated plates and incubated at 37°C for 1 h, followed by incubating with HRP conjugated monoclonal anti-His (1:1000 dilution with blocking buffer). Absorbance at 450 nm was measured and compared. Samples were considered positive when the OD value was over 0.15 after subtracting the background.

Besides, in contrast to anti-preS1 that could recognize only L protein in serum, polyclonal anti-preS was able to capture both L and M proteins present in patient's serum (Fig. 3). No S protein could be detected by polyclonal anti-preS, while it can be obviously detected by monoclonal anti-S as expected.

**Figure 3:** Polyclonal anti-preS recognizes both L and M protein. Western blot analysis was performed using polyclonal anti-preS, and monoclonal anti-S, respectively. The bands that recognized by polyclonal anti-preS correspond to the large protein (p39/gp42) and M protein (gp33/gp36) [41]. Monoclonal anti-S used as a positive control could detect the S protein (p24/gp27) in addition to the L and M proteins.

### Detection of HBsAg and HBpreSAg in sera from hepatitis B patients

HBsAg in sera from 50 HBeAg positive and 104 HBeAg negative (anti-HBe positive) HBV patients had been quantitated (Fig. 4). The average value of HBsAg was higher (p = 0.995) in HBeAg positive HBV patients (24.0 ± 19.4 μg/ml) than that of HBeAg negative patients (1.70 ± 2.16 μg/ml). Twenty serum samples of healthy people with normal liver functions and without any clinical marker of HBV infection were used as controls and no HBsAg and HBpreSAg can be detected.

**Figure 4:** The presence of HBpreSAg in serum of HBV patients and its correlation with HBsAg. The rate of HBpreSAg presence in serum of HBeAg-negative patients and HBeAg-positive patients were shown in (A) and (C), respectively. The white bars represent HBpreSAg negative patients and the black bars represent HBpreSAg positive patients. Correlation of HBpreSAg levels with HBsAg levels in serum of HBV patients were indicated in (B) for HBeAg-negative patients and (D) for HBeAg-positive patients. The X axis indicates the serum HBsAg content and the Y axis is the absorbance of the HBpreSAg ELISA test at 450 nm after background correction.

Detection of HBpreSAg by ELISA was carried out using the same serum samples. In order to ensure HBsAg levels below 20 μg/ml, samples were diluted by 2X and 10X for HBeAg-negative patients and HBeAg-positive cases, respectively. All samples were tested in duplicate and the average OD_450 _was taken. In the 104 HBeAg-negative HBV patients, 55 (53%) were HBpreSAg negative and 49 (47%) were positive, while in the 50 HBeAg positive HBV patients, 35 (70%) were HBpreSAg positive and 15 (30%) were negative. The average OD_450 _values of HBpreSAg in patients from the two groups were also distinct (p = 0.87), which was 0.62 ± 0.54 for the HBeAg positive patients and 0.35 ± 0.23 for HBeAg negative patients.

These results suggested that levels of both HBsAg and HBpreSAg were apparently higher in HBeAg-positive patients. Serial dilutions were performed on serum samples to compare the relative amount of HBpreSAg in both groups. The result showed that HBpreSAg of about 50% of the samples from HBeAg positive patients were still detectable after 50 fold dilution. A two-fold dilution of the serum samples from HBeAg negative patients gave a similar result.

### Correlation of Ag with HBsAg

The serum level of HBpreSAg was compared with that of HBsAg (Fig. 4A,4C). The HBpreSAg positive portion increased with HBsAg in both groups. However, HBpreSAg and HBsAg presented different relationships in the two groups. The correlation efficiency between HBpreSAg and HBsAg is 0.713 (p < 0.01), which indicated a liner correlation between HBsAg and HBpreSAg for HBeAg positive patients (Fig. 4D), which is not distinctly linear in HBeAg negative patients (Fig. 4B).

### Correlation of HBpreSAg with HBeAg

For the 50 HBeAg-positive patients, the levels of HBpreAg and HBeAg were compared and the result showed no clear quantitative correlation (data not shown).

### Correlation between HBpreSAg and serum HBV DNA copies

Among the 50 HBeAg-positive patients detected, 43 patients showed HBV DNA positive and 35 showed HBpreSAg positive. In twelve HBV DNA positive cases, HBpreSAg could not be detected. In four HBpreSAg positive patients HBV DNA was below the detection limit by PCR. For the patients showed positive in both HBpreSAg and HBV DNA, the correlation efficiency between HBpreSAg and HBV DNA was 0.83 (p = 0.01), suggesting a positive correlation (Fig. 5A).

**Figure 5:** Correlation of HBpreSAg levels with HBV DNA copies in serum of HBeAg positive patients (A) and HBeAg negative (anti-HBe positive) patients (B). (A) The X axis indicates the average HBV DNA copies at different levels and the Y axis indicates the average absorbance of the HBpreSAg ELISA test at 450 nm corresponding to the different HBV DNA levels. (B) The detection rate of HBV DNA was analyzed at different levels of HBpreSAg present in serum as shown in the left panel. The rates of HBV DNA positives and negatives at each HBpreSAg level are shown at the top of each vertical bar. The white bars represent the number of HBV DNA negative patients and the black bars represent that of HBV DNA positive patients. The detection rate of HBpreSAg present in serum was analyzed at different levels of HBV DNA as shown in the right panel. The rates of HBpreSAg positives and negatives at each HBV DNA level are shown at the top of each vertical bar. The white bars represent the number of HBpreSAg negative patients and the black bars represent that of HBpreSAg positive patients.

Among the 104 HBeAg-negative patients studied, the HBV DNA copies of 99 patients have been examined. Only 28 (28%) patients showed positive HBV DNA level, of which 17 cases were HBpreSAg positive. In the remaining patients, 41showed levels of both HBpreSAg and HBV DNA below their detection limits. In addition, 30 of HBV DNA negative patients were tested as HBpreSAg positive. The portion of HBpreSAg positive increased obviously with HBV DNA copies (Fig. 5B). Analysis of the levels of HBpreSAg and HBsAg between HBV DNA negative and positive patients in HBeAg-negative group also showed an obvious difference (p-value was 0.998 for HBsAg and 0.95 for HBpreSAg). In HBV DNA negative patients, the averages of HBsAg and HBpreSAg were 1.4 ± 1.9 ug/ml and 0.29 ± 0.43 (OD450), while for the HBV DNA detectable patients the average was 2.3 ± 2.5 μg/ml and 0.43 ± 0.53 μg/ml (OD450), indicating that HBsAg and HBpreSAg were correlated well with HBV DNA copies.

### Follow up study

Among the 23 HBeAg positive and anti-HBe negative patients enrolled in the follow up study, 19 showed an obvious decrease in HBpreSAg levels after IFN-α treatment. None of the patients on therapy became HBsAg negative (<0.01 μg/ml) even though their HBsAg levels decreased (Fig. 6).

**Figure 6:** Changes of HBpreSAg levels and other serologic markers of the three Types patients for follow up study. Black square represents HBpreSAg (OD_450_), black triangle represents HBsAg (OD_450_), white circle represents ALT (IU/l) and white triangle represents HBV DNA copies (copies/ml). A typical sample for Type I-III was shown. (A) The levels of HBpreSAg, HBsAg, ALT and HBV DNA decreased significantly without rebound in Type I patients. (B) Type II patients responded to the IFN-α treatment well initially but rebounded at the end check point. (C) Type III patients did not respond well to the IFN-α treatment.

Since HBV DNA copies are generally considered as the measure of viral loads, the response patterns of the 23 patients after IFN-α therapy were divided into three types based on the reduction pattern of HBV DNA copies (Fig. 6, Table 1). The pattern of HBpreSAg and other serological markers were analyzed within each group.

**Table 1:** Average changes of HBpreSAg and HBV DNA after IFN treatment and comparisons of different HBV markers.

	DNA^a ^(0 wk)	DNA^a ^(0/24 wk)	DNA^a ^(0/48 wk)	HBpreSAg (0 wk)	HBpreSAg (0/24 wk)	HBpreSAg (0/48 wk)	ALT (0 wk)
Average (type I)	8.3	1.9	3.7	0.7	1.7	2.2	379
Average (type II)	8.1	2.8	-0.4	0.9	3.3	1.9	327
Average (type III)	8.5	0.2	0.5	0.8	1.2	1.5	423

(0/24 wk) and (0/48 wk) present the reduction of HBV DNA (logs) or HBpreSAg (folds) at 24 week and 48 week respectively compared to that of the beginning point. ^a^HBV DNA copies were presented in logarithm.

In type I group (Fig. 6), at the end point of the follow up (48 weeks), HBV DNA copies dropped by about 3-logs. HBeAg seroconversion was observed. The outcome for this group after IFN-α therapy should be considered as remission based on viral load reduction. The reduction of the HBpreSAg levels was significant in most cases and the levels of HBsAg decreased to a similar extent. The serum alanine aminotransferase (ALT) levels of four of the five patients showed an obvious decrease during IFN-α treatment, and below the limit of normal at the end check point.

In type II group (Fig. 6), based on the reduction of HBV DNA copies, seven patients responded to the IFN-α treatment well initially by the end of 24 weeks, but their viral loads rebounded to high levels at the end point. The pattern of HBpreSAg changes was similar to that of HBV DNA copies in this group, 3.3-fold reduction on average at 24 weeks and rebounded to 1.9-fold reduction at 48 weeks (Table 1). Four patients' anti-HBe was observed as positive during the IFN-α treatment but returned to negative later. An obvious drop of the ALT level was observed after IFN-α treatment, but which rebounded at the last check point in five of the seven patients.

In type III group (Fig. 6), 11 patients did not show any significant reduction in their viral loads during IFN-α treatment. The level of HBpreSAg decreased slightly following the IFN-α treatment. The level of HBsAg remained high mostly and their HBeAg remained positive through the course of treatment. Changes of ALT levels showed similar pattern.

As shown in Table 1, the average values of viral load reduction and HBpreSAg reduction were calculated for each group described above. ALT levels at the beginning of the treatment were also presented. The HBpreSAg levels were reduced relatively more in type I and II groups than in type III group.

## Discussion

### preS antigen is a potential significant serological marker for chronic hepatitis B virus infection

Full length preS is exclusively present in the large protein (L) and has been shown to be associated with virus attachment to the host cell receptor and membrane fusion during entry [20]. Since preS mainly exist in the DNA-containing Dane HBV particles, detection of HBpreSAg present in serum of HBV patients may have a clinical value in management of HBV infection. In previous reports, radioimmunoassays using monoclonal antibodies have been used to detect HBsAg, preS1 or preS2 antigen in the sera of HBV patients respectively, and these assays were proved to have well-defined specificities[15,17,21]. However, using antibodies against full length preS including both preS1 and preS2 to detect the serum preS has not been reported so far.

In this study, we have established a double antibody sandwich ELISA system that could capture both L protein and M protein in order to reflect the full presence of HBpreSAg in serum of HBV patients (Fig. 3). Since functional three dimensional structure formed from the full length of preS is the structure basis for displaying epitopes and detecting active Dane viral particles, using antibodies against a well folded preS can result in a more sensitive detection of preS antigen in serum. However, high levels of HBsAg in sera may still introduce a bias in HBpreSAg measurements. This problem was circumvented by diluting serum samples to ensure HBsAg below 20 μg/ml, the standard that brought no interference into assay of HBpreSAg as demonstrated by our experiment. Therefore, both sensitivity and specificity of our ELISA were greatly improved in comparison with other forms of HBpreSAg tests.

Our results indicate that HBpreSAg correlated well with HBV DNA copies in serum. These results are consistent with the results of Petit's[17,21] and Garbuglia's[22]. One difference is that Petit's data showed that PCR was an adequately sensitive method that could detect HBV DNA in roughly half of the HBpreSAg negative sera, while this ratio is 21% in our study. Of the 47 HBpreSAg positive patients in this study, 30(64%) had no detectable HBV DNA, which was consistent with the result of Alberti's observation. Their results showed that preS1 and preS2 could also been detected from 7 out of 10 cases (70%) with no evidence of viral replication, in addition to HBV DNA positive cases[23]. Our observations and Alberti's indicated that in the serum of HBV patients, especially for the HBeAg-negative patients, preS is another significant serological marker for active HBV infection in addition to HBV DNA.

Both HBeAg and HBV DNA copies are commonly used as clinical markers of active HBV replication, and treatments are recommended based on diagnostic tests of these markers. Our results indicate that HBpreSAg could be another valuable marker to supplement HBeAg (Table 2). When HBpreSAg was compared to HBV DNA copies, the sensitivity was 68% (CI, 95%, 55–78), and the specificity was 56% (CI, 95%, 45–67). This gives an overall accuracy of 62% of our HBpreSAg test. By the same comparison, the sensitivity of the HBeAg test was 61% (CI, 95%, 48–72), and the specificity was 91% (CI, 95%, 82–96), leading to an overall accuracy of 77%. Similar results are obtained when HBpreSAg is compared to HBeAg. These results suggest that HBpreSAg can serve as a serological marker for HBV replication with sensitivity slightly higher than that of HBeAg. However, the overall accuracy of the HBpreSAg test was dampened due to a low specificity, but not too much off compared to the HBeAg test (62% versus 77%). If the results of HBV DNA are reconciled with those of HBeAg assuming that the case was truly positive if HBV DNA and HBeAg were positive for HBpreSAg+ cases, and the case was truly negative if HBV DNA and HBeAg were negative for HBpreSAg- cases, the sensitivity, the specificity, and the overall accuracy of the HBpreSAg test would be, 81%, 65%, and 72%, respectively (Table 3). This observation argues that a HBpreSAg test would be valuable for detecting HBV replication in HBV patients and suggests further improvements of the HBpreSAg test.

**Table 2:** Comparisons of serological markers for HBV replication versus HBVDNA copies in serum specimens.

	HBV DNA+	HBV DNA-		Sensitivity(%)	Specificity(%)	PPV(%)	NPV (%)	Overall (%)
HBpreSAg+	48	34		68	56	59	66	62
HBpreSAg-	23	44	CI,95%	55–78	45–67			
n = 149								

	HBV DNA+	HBV DNA-		Sensitivity(%)	Specificity(%)	PPV(%)	NPV (%)	Overall (%)
HBeAg+	43	7		61	91	86	72	77
HBeAg-	28	71	CI,95%	48–72	82-96			
n=149								

	HBeAg+	HBeAg-		Sensitivity(%)	Specificity(%)	PPV(%)	NPV (%)	Overall (%)
HBpreSAg+	35	49		70	53	42	79	58
HBpreSAg-	15	55	CI,95%	55-82	43-63			
n=154								

**Table 3:** Comparison of the HBpreSAg test versus HBV DNA copies in serum specimens, with reconciliation by HBeAg results.

	HBV+ (DNA+ reconciled by HBeAg+)	HBV- (DNA- reconciled by HBeAg-)		Sensitivity(%)	Specificity(%)	PPV(%)	NPV (%)	Overall (%)
HBpreSAg+	52	30		81	65	63	82	72
HBpreSAg-	12	55	CI,95%	72-89	58-70			
n=149								

### Potential application of HBpreSAg in IFN-α treatment

Interferon-α, as an approved treatment for hepatitis B, has been widely used in clinical therapy[4,24-33]. According to previous reports, the levels of serum HBV DNA, HBsAg, HBeAg and other serological markers decrease during the IFN-α treatment if the patient responded positively to the IFN-α therapy. Long-term follow up studies showed that most responders maintained their responses though very few people had complete eradication of HBV[31]. To date, there lacks study to follow the serum levels of full length preS in response to IFN-α treatment.

The second objective of this study was to monitor the change of HBpreSAg in sera of the chronic hepatitis patients before, during and after IFN-α treatment, to investigate the correlation of HBpreSAg with HBV DNA copies and HBsAg. The result showed that the level of HBpreSAg varied in different sera. The change in HBsAg levels, HBV DNA copies, ALT levels, and HBpreSAg levels had similar patterns in most cases, which is similar to the result of Taliani et al's[34]. This observation is consistent with the idea that HBpreSAg was elevated when HBV started active replication, suggesting that preS is correlated to other serological markers to a certain extent but has its own merit as discussed below, and could serve as an alternative serological marker.

Another interest was to identify any potential predictor that could classify types of patients' response to IFN therapy. According to the variation of viral loads, the 23 patients could be divided into three groups: sustained responders, responders with rebound, and non-responders. The reduction of serum HBpreSAg levels was comparatively more pronounced in type I and II than in type III (Table 1). This result indicated that patients with a significant reduction of HBpreSAg were inclined to have a better response to IFN treatment despite high copies of HBV DNA. More rapid HBV DNA reduction right after the treatment in type II than type I also demonstrated this point. Meanwhile, more rapid reduction of HBpreSAg in type II than that of type I may suggest more active replication of HBV in type II, which could explain the rebound occurred in this type after 24 week treatment. With the relative high level of ALT at the end point for the type II group, the patients may require further treatment. A combination therapy of IFN and nucleosides should be considered to improve outcome as shown by Chan et al. [35] or the IFN treatment should be extended.

Patients with high ALT and low HBV DNA are inclined to respond well to interferon treatment [36-38]. In our study, this phenomenon was also observed and its pattern was similar to that of HBpreSAg (Table 1).

Though there is no clear reason for the prediction of IFN treatment based on ALT, HBV DNA or HBpreSAg, our study revealed a potential application of HBpreSAg in prediction of IFN treatment. Moreover, this experiment revealed that the reduction rate of HBpreSAg appeared to be a predictor for the outcome of interferon treatment and perhaps HBpreSAg was involved in interplays between interferon activities and HBV virus infection, which, however, required further investigation by examining more patients.

## Conclusion

The establishment of the new ELISA method enables us to capture both the L and M proteins, and properly reflect the full presence of HBpreSAg in serum of HBV patients. Applying this assay to serum samples from HBeAg-negative patients, 30 out of 47 HBpreSAg positive patients showed no evidence of viral replication. HBpreSAg can serve as a serological marker for HBV replication with sensitivity slightly higher than that of HBeAg. The follow up study showed that HBpreSAg levels in sera of the chronic hepatitis patients examined during and after IFN-α treatment changed in similar patterns, in most cases, with HBsAg levels, HBV DNA copies and ALT levels. More importantly, reduction of HBpreSAg levels indicated a good response to IFN-α treatment and vice versa, suggesting the level of HBpreSAg in conjunction with the HBV DNA copies might be a potential predictor of treatment efficacy. Limited by the number of patients, a reliable statistical analysis could not be conducted among the three types of patients. However, the potential of HBpreSAg and HBV DNA in predicting IFN-α treatment is well presented in this study. Detection of full presence of HBpreSAg in this study provided an alternative serological marker and will allow for an improved evaluation of chronic HBV infection.

## Methods

### Sera

The patients with clinical evidence of hepatitis B from People's Hospital of Peking University were chosen in this study. Sera from 104 HBeAg-negative (anti-HBe positive) chronic hepatitis B and 50 HBeAg-positive outpatients with identified age and gender have been tested. Sera of 20 healthy people without any clinical markers of HBV infection and with normal liver functions were used as negative control. 23 inpatients tested HBeAg positive and anti-HBe negative were enrolled in a 48 week follow-up study with 3 MU IFN-α thrice weekly applied in the beginning 24 weeks. Their serum specimens were collected at 5 check points at twelve week intervals, and their HBpreSAg, HBV-DNA, HBsAg, HBeAg and ALT were analyzed as well. All samples were collected according to the guidelines of the ethical committee in Peking University People's hospital with patients' written consent.

### Preparation and examination of anti-preS polyclonal antibody

A polyclonal antiserum to preS was prepared by immunizing rabbits with purified full length preS protein containing both preS1 and preS2 (≥95% purity, Fig. 1A) of subtype adw (Accession No. P03142) following our previous procedure[39]. Western blot was carried out to test both the specificity of polyclonal anti-preS using recombinant preS protein and the ability of polyclonal anti-preS in detecting both preS1 and preS2 regions in patient's serum.

### Detection of HBpreSAg in serum by a double antibody sandwich ELISA

preS antigen was determined in serial serum samples using a double antibody sandwich ELISA with polyclonal anti-preS generated as described above and monoclonal anti-HBs (raised by immunizing mice with purified virus particles) as follows. Four serial dilutions of sera (1:2, 1:10, 1:50 and 1:250 diluted with blocking buffer in PBS, pH7.4) were added to anti-preS coated wells and incubated at 37°C for 1 h. The wells were then incubated with HRP conjugated monoclonal anti-S (1:1000 dilution with blocking buffer containing 3% BSA, 20% goat serum in PBS). Absorbance at 450 nm was measured by microplate reader (Prolong, China). Samples were considered positive when the OD value was over 0.15 after subtracting the background.

### Detection of HBsAg in serum of chronic HBV patients

HBsAg was determined in the same serum samples by using an ELISA kit (Wan Tai Diagnostics Corp, Beijing, China), following the manufacturer's instructions. Four serial dilutions of sera (1:20, 1:100, 1:500 and 1:2500 diluted with blocking buffer in PBS, pH7.4) were applied and absorbance at 450 nm was measured. In order to quantify HBsAg in sera, known amount of recombinant S protein (Fudan-Yueda Bio-Tech Co. China) was serially diluted to plot a standard curve by using the same ELISA kit.

### Detection of HBeAg in serum of chronic HBV patients

Serum HBeAg measurements were performed based on an immunoenzymometric assay (IEMA) using HBeAg/Ab IEMA Well (RADIM S.pA., Italy) according to the manufacturer's instruction.

### Quantification of HBV DNA in serum by PCR

Quantification of serum HBV DNA was performed by the LightCycler PCR system (Roche, Basel, Switzerland) using fluorescent quantitative PCR kits (PG Biotech, Shenzhen, China). The sensitivity of the assay was 300 copies/ml of HBV DNA.

### Serum alanine aminotransferase (ALT) measurements

Serum ALT measurements were performed with the Reflotron system (Fa. Boehringer Mannheim). [40] The upper normal range of ALT was 40 IU/l and this threshold was given by the manufacture.

## Abbreviations

HBV, hepatitis B virus; HBsAg, hepatitis B surface antigen; HBpreSAg, hepatitis B pre-surface antigen; HBeAg, hepatitis B e antigen, anti-HBs, antibody to HBsAg; anti-preS, antibody to hepatitis B preS antigen; IFN-α, interferon-alpha; ALT, alanine aminotransferase.

## Competing interests

The author(s) declare that they have no competing interests.

## Authors' contributions

ML – carried out protein purification, performed ELISA analysis and assisted with manuscript preparation. XZ – prepared polyclonal anti-preS, interpreted the data, and assisted with manuscript preparation. LW – provided patients sera, measured HBV DNA and ALT. SQ – constructed the protein expression vector. TZ – assisted in study design and provided monoclonal anti-HBs antibody. LL – assisted in ELISA analysis. XG – assisted in study design and helped edit the manuscript. ML – designed and oversaw the study, interpreted the data and wrote the manuscript. XZ -designed and oversaw the study, interpreted the data and wrote the manuscript. All authors read and approved the final manuscript.
